# Parameter Tuning of PID Controller for Beer Filling Machine Liquid Level Control Based on Improved Genetic Algorithm

**DOI:** 10.1155/2021/7287796

**Published:** 2021-07-23

**Authors:** Liqing Xiao

**Affiliations:** School of Mechanical and Electrical Engineering, Huainan Normal University, Huainan 232038, China

## Abstract

Parameter tuning of PID controller for liquid level control of beer filling machine was studied in this paper, which can meet the demand of accurate controlling in beer production and improve the rapidity under the same conditions. Firstly, an improved genetic algorithm was proposed which has been verified by eight kinds of test functions. Simulation results revealed that, in comparation with other modified particle swarm optimization algorithm and modified genetic algorithm, the algorithm proposed in this work is not only capable to improve the convergence speed and precision under the same experimental conditions but also to improve the probability to converge to the optimal value. Finally, the proposed algorithm was applied to the parameter tuning of the PID controller of beer filling machine for liquid level control. Superior property had been obtained, which implied an effective improvement in the rapidity with the premise of steady-state error exclusion.

## 1. Introduction

Usually, in order to improve the performance of the control systems, various measures need to be taken [1, 2]. PID controller has been widely employed in control systems due to its basal principle, excellent robustness, and considerable reliability [3–7]. Nevertheless, the controlling performance of PID controller relies on the value selection of scale coefficient, integral coefficient, and differential coefficient. With the purpose to improve the performance of the control system as possible, the parameter tuning of PID controller has become one of the research hotspots currently [8–10].

The quantization factor and scaling factor were iteratively optimized in the offline state by using particle swarm optimization algorithm approach to adjust the fuzzy PID parameters rapidly, and the control system was simulated and analyzed by MATLAB, which has been reported in pervious literature [11]. Furthermore, Gao et Al. proposed a new objective function construction method according to the control system overshoot based on the conventional genetic algorithm to realize the parameter optimization of PID [12]. As presented in literature [13], aiming to overcome the shortages of the traditional quantum genetic algorithm, Jian-xin FENG et al. had addressed the premature problem of the traditional quantum genetic algorithm and improved the convergence speed through the following five aspects including coding method, population initialization, quantum revolving gates, quantum mutation, and the increase of quantum catastrophe. The optimized algorithm presented above had been applied to the parameter optimization of fuzzy self-tuning PID controller. Moreover, in order to deal with the complexity of parameter tuning of the fractional-order PID controller, Su WANG et al. had introduced the chaotic perturbation into the Beetle Antennae Search algorithm and promoted a parameter tuning approach of fractional-order PID controller to enhance optimization performance of algorithm according to the random perturbation of individual positions resulted from the logistic mapping formula [14]. As known that, BAS had been challenged by the local optimum and low precision due to its prematurity, Shijiao SHAN et al. had integrated the efficient BAS algorithm with the traditional bat algorithm and used it for the PID parameter optimization to achieve a faster response [15]. In addition, aiming at the problem of oscillation caused by excessive selection of learning rate in the learning process of the traditional BP neural network, Huangshui HU et al. had proposed a new adaptive tuning algorithm for PID parameters of BP neural network to alleviate the oscillation phenomenon effectively and accelerate the convergence speed of the algorithm [16].. The convergence speed and stability of the genetic algorithm were improved in literature [17] to realize the online adjustment of PID control parameters with the optimized initial weight of BP neural network employed. Liu and Chen [18] presented tuned PID parameters with high convergence accuracy and fast convergence speed by using cellular genetic algorithm (CGA). Cao and Feng [19] designed an adaptive fuzzy PID controller based on particle swarm optimization algorithm according to the urban rail train braking model. Ye [20] improved the searching ability of the particle swarm optimization algorithm by adjusting the adaptive inertia factor, which has been applied to adjust the PID parameters of the temperature control system of injection molding machine online and further improve the control accuracy. Considering the limitations of the conventional PID controller, Zhao and Fu proposed a scheme combining the fuzzy system and BP neural network [21]. Meanwhile, whale optimization algorithm (WOA) was adopted for further optimization in the improvement of dynamic performance and steady-state accuracy of the control system.

## 2. Improved Genetic Algorithm

The improved genetic algorithm refers to the random division of variable interval according to the setting interval number, while the initial population is generated according to the fitness value of the midpoint of the interval and roulette wheel selection. In the iterative process of the algorithm, the PSO algorithm was introduced into the crossover operation according to the probability. The individual with the lowest fitness value would be substituted by random individuals generated via the same method in developing the population.

### 2.1. Flow Diagram of Improved Genetic Algorithm

Step 1: setting the parameters in the improved genetic algorithm, including population numbers, interval numbers, maximum iterations, crossover probability, mutation probability, introduction probability of particle swarm optimization algorithm, learning factor, maximum inertia weight, minimum inertia weight, allowable error, etc.
Step 2: dividing the variable intervals randomly according to the interval number settings in Step 1 and substituting the midpoint of the intervals into the fitness function of the algorithm to estimate the fitness value. On this basis, according to the algorithm parameters set in Step 1 and the roulette selection, the initial population of the algorithm has been generated.
Step 3: calculating the fitness value of each individual among population to evaluate each individual and to complete the selection operation.
Step 4: executing the crossover operation according to the crossover probability and the introduction probability of the particle swarm optimization algorithm which has been set in Step 1. The particle swarm optimization algorithm updates the speed and position abiding to equation (1).
  (1) $$\begin{array}{c} \left\{\begin{array}{c} V_{i}^{k+1}=\omega \times V_{i}^{k}+c_{1}\times \text{rand }1\times \left(pbest_{i}-X_{i}^{k}\right)+c_{2}\times \text{rand }2\times \left(gbest_{g}-X_{i}^{k}\right),\\ X_{i}^{k+1}=X_{i}^{k}+V_{i}^{k+1}, \end{array}\right. \end{array}$$
where the optimum algorithm population, global optimum, speed, and position of population size were denoted as **pbest**_*i*_, **gbest**_*g*_, **V**, and **X**, respectively. *k* referred to the iterations of the improved genetic algorithm, while *c*_1_ and *c*_2_ referred to the learning factors. rand 1 and rand 2 represented the random numbers uniformly distributed within (0, 1).
The inertia weight has been labeled as *ω*, which diminished with four different strategies associated to the probability to enhance the optimization ability during the iterative process in improved genetic algorithm, as revealed in equations (2)–(5) [22].
  (2) $$\begin{array}{c} \omega =\omega_{\max}-\frac{\text{era}}{\max e}\cdot \left(\omega_{\max}-\omega_{\min}\right), \end{array}$$
  (3) $$\begin{array}{c} \omega =\omega_{\min}+\left(\omega_{\max}-\omega_{\min}\right)\cdot {\left(\frac{\max e-\text{era}}{\max e}\right)}^{2}, \end{array}$$
  (4) $$\begin{array}{c} \omega =\omega_{\min}+\left(\omega_{\max}-\omega_{\min}\right)\cdot {\left(\frac{\max e-\text{era}}{\max e}\right)}^{3}, \end{array}$$
  (5) $$\begin{array}{c} \omega =\omega_{\min}+\left(\omega_{\max}-\omega_{\min}\right)\cdot {\left(\frac{\max e-\text{era}}{\max e}\right)}^{4}. \end{array}$$
The maximum and minimum of inertia weights were marked as *ω*_max_ and *ω*_min_, where max*e* and era represented the maximum and the current number of iterations in the improved genetic algorithm, respectively.
Step 5: executing mutation operation according to the mutation probability set in Step 1.
Step 6: calculating the fitness value for each individual in population and generating a random individual with the same method in generating the initial population of the algorithm described in Step 2, which would be used to substitute the individual with the lowest fitness value at present.
Step 7: determining whether the termination condition of the algorithm has been met based on the number of iterations and the allowable error of the algorithm. And the algorithm would terminate or skip to Step 3 for cyclic calculation.

### 2.2. Experimental Results of Improved Genetic Algorithm

In order to verify the performance under the same experimental conditions, the improved genetic algorithm had been applied to the optimization of eight different kinds of typical test functions. The simulation experimental environment is MATLAB R2009 B version, in which numbers including 50 in the population of the algorithm, 12 in the number of intervals, 200 in the maximum number of iterations, 0.90 in the crossover probability, 0.01 in the mutation probability, 2 × 10^−15^ in the allowable error, 0.5 in the introduction probability of particle swarm optimization algorithm, and 0.90 and 0.10 in the maximum and minimum inertial weight, respectively, had been set. Different algorithms had been run 100 times each.

The expressions of the eight kinds of test functions had been demonstrated in equations (6)–(13), and corresponding function images are given in Figure 1. The average convergence curves of different algorithms are presented in Figure 2 with the average convergence precision of different algorithms shown in Table 1. The average convergence algebras and the probabilities of convergence to the optimal value are compared in Tables 2 and 3 .

(6) $$\begin{array}{c} f\left(x_{1},x_{2}\right)=-20e^{-\left(\sqrt{\left(1/2\right)x_{1}^{2}+\left(1/2\right)x_{2}^{2}}\right)/5}-e^{\left(\cos\left(2\pi x_{1}\right)+\cos\left(2\pi x_{2}\right)\right)/2}+20+e,\;x_{i}\in \left[-50,50\right], \end{array}$$

(7) $$\begin{array}{c} f\left(x_{1},x_{2}\right)=\left|x_{1}\sin\left(x_{1}\right)+0.1x_{1}\right|+\left|x_{2}\sin\left(x_{2}\right)+0.1x_{2}\right|,\;x_{i}\in \left[-20,20\right], \end{array}$$

(8) $$\begin{array}{c} f\left(x_{1},x_{2}\right)={\left(x_{1}x_{2}-x_{1}+1.5\right)}^{2}+{\left(x_{1}x_{2}^{2}-x_{1}+2.25\right)}^{2}+{\left(x_{1}x_{2}^{3}-x_{1}+2.625\right)}^{2},\;x_{i}\in \left[-30,30\right], \end{array}$$

(9) $$\begin{array}{c} f\left(x_{1},x_{2}\right)=x_{1}^{2}+2x_{2}^{2}-0.3\;\cos\left(3\pi x_{1}\right)-0.4\;\cos\left(4\pi x_{2}\right)+0.7,\;x_{i}\in \left[-80,80\right], \end{array}$$

(10) $$\begin{array}{c} f\left(x_{1},x_{2}\right)={\left(x_{1}^{2}-1\right)}^{2}+{\left(x_{2}^{2}-2\right)}^{2},\;x_{i}\in \left[-70,70\right], \end{array}$$

(11) $$\begin{array}{c} f\left(x_{1},x_{2}\right)=7x_{1}^{2}-6\sqrt{3}x_{1}x_{2}+13x_{2}^{2},\;x_{i}\in \left[-60,60\right], \end{array}$$

(12) $$\begin{array}{c} f\left(x_{1},x_{2}\right)=1-\cos\left(2\pi \sqrt{x_{1}^{2}+x_{2}^{2}}\right)+0.1\sqrt{x_{1}^{2}+x_{2}^{2}},\;x_{i}\in \left[-20,20\right], \end{array}$$

(13) $$\begin{array}{c} f\left(x_{1},x_{2}\right)=0.5+\frac{\sin^{2}{\left(x_{1}^{2}-x_{2}^{2}\right)}^{2}-0.5}{1+0.001{\left(x_{1}^{2}+x_{2}^{2}\right)}^{2}},\;x_{i}\in \left[-80,80\right]. \end{array}$$

Among them, the improved genetic algorithm proposed in this paper was presented as algorithm 1, while algorithm 2 was the modified particle swarm optimization algorithm based on interval algorithm and modified elite strategy, and algorithm 3 belonged to the improved genetic algorithm promoted in literature [22].

As revealed from Tables 1–3, with the same parameter settings in eight different test functions, the average convergence values of algorithm 1, algorithm 2, and algorithm 3 were 1.008 × 10^−11^, 4.9460 × 10^−2^, and 4.3543 × 10^−2^ with the average convergence algebras of 77, 155, and 159 and average probability of converging to the optimal value of 98.8750%, 61.7500%, and 59.3750%, respectively.

It is concluded that compared with algorithms 2 and 3, the improved genetic algorithm proposed in this paper improves the convergence accuracy, the convergence speed, and the probability of convergence to the optimal value of algorithm effectively, which is also implied in Figure 2.

## 3. Parameter Tuning of PID Controller for Liquid Level Control of Beer Filling Machine

### 3.1. Mathematical Modelling

Considering of the balance between inflow and outflow volume of liquid, the height of liquid level (*H*), the cross-sectional area of the liquid storage tank (*A*), and the inflow (*Q*_1_) and outflow (*Q*_2_) liquid obey the equation as follows [23, 24]:

(14) $$\begin{array}{c} A\frac{\text{d}H}{\text{d}t}=Q_{1}-Q_{2}, \end{array}$$

which can be rewritten in the following form of increment:

(15) $$\begin{array}{c} A\frac{\text{d}\Delta H}{\text{d}t}=\Delta Q_{1}-\Delta Q_{2}. \end{array}$$

To simplify the mathematical model of the control system, we assumed that the outflow increment was proportional to the liquid level increment and was inversely proportional to the valve resistance of the load valve, which has been shown in the following equation [23, 24]:

(16) $$\begin{array}{c} \Delta Q_{2}=\frac{\Delta H}{R_{2}}. \end{array}$$

Based on equations (14) and (16),

(17) $$\begin{array}{c} RA\frac{\text{d}\Delta H}{\text{d}t}+\Delta H=R\Delta Q_{1}. \end{array}$$

By using Laplace transformation, we get

(18) $$\begin{array}{c} G\left(s\right)=\frac{H\left(s\right)}{Q_{1}\left(s\right)}=\frac{R}{RAs+1}=\frac{K}{Ts+1}. \end{array}$$

Considering the hysteresis of liquid level changes in realistic engineering problems, the liquid level control system can be approximately seen as a first-order inertial hysteresis system with the transfer function shown in the following equation [23, 24]:

(19) $$\begin{array}{c} G\left(s\right)=\frac{H\left(s\right)}{Q_{1}\left(s\right)}=\frac{K}{Ts+1}e^{-\tau s}, \end{array}$$

where *K*, *T*, and *τ* are defined as 5, 160, and 3 in this paper.

### 3.2. Stability Analysis of Control System

Stability laid the foundation for the operation of the control system. Hence, it is a priority to determine the stability of a certain control system. Since the control system consisted of a nonlinear delay part, the analysis of stability has to be realized via the observation of the unit step response curves and calculation of the amplitude and phase angle margin of a control system, instead of the Routh–Hurwitz stability criterion. The unit step response curve of the control system is shown in Figure 3, and the Bode diagram is shown in Figure 4.

Figure 3 illustrates the convergence in unit step response curve of the control system. The amplitude margin of the control system (24.5 dB) and the phase angle margin (96.3°) were both larger than zero, as shown in Figure 4, which confirmed the stability of the control system.

### 3.3. Parameter Tuning of PID Controller

In order to improve the performance of the control system, algorithms 1, 2, and 3 have been employed to correct PID controller parameters, and the fitness function is shown in the following equation:

(20) $$\begin{array}{c} F\left(X\right)=\frac{1}{t_{s}+10\times \sigma \%}P\left(X\right), \end{array}$$

where *X* represented the variate of proportional coefficient (*K*_*P*_), integral coefficient (*K*_*I*_), and differential coefficient (*K*_*D*_) of the PID controller. *t*_*s*_, *σ*% were denoted as the adjustment time and overshoot of the control system, respectively. *P*(*X*) referred to the penalty function. Thus, the expression is shown in the following equation:

(21) $$\begin{array}{c} P\left(X\right)=\left\{\begin{array}{cc} 1, & \text{if }\left|e_{\text{ss}}\right|<10^{-10},\\ 0, & \text{if }\left|e_{\text{ss}}\right|\geq 10^{-10}, \end{array}\right. \end{array}$$

where *e*_ss_ is the steady-state error of the control system.

The convergence curves of algorithms 1, 2, and 3 are presented in Figure 5.  Figure 6 shows the unit step response curves of the control system corresponding to the optimal results. Performance indexes of the control system are shown in Table 4.

The steady-state error (*e*_ss_) of the control system had been eliminated effectively and the adjustment time (*t*_*s*_) of the control system was reduced after PID correction, which were elucidated in both Figure 6 and Table 4. Moreover, among these three types of algorithms, algorithm 1 had been proved to have the most remarkable performance in this paper.

However, it also caused a large oscillation which was responsible for a large overshoot. Moreover, fitness function presented in equation (22) can be applied to improve the stability of the control system.

(22) $$\begin{array}{c} F\left(X\right)=\frac{1}{\sigma \%}P\left(X\right). \end{array}$$

Maintaining the simulation experimental environment and algorithm parameters, the convergence curves of algorithms 1, 2, and 3 are provided in Figure 7. The unit step response curves of the control system corresponding to the optimal results are shown in Figure 8.

The overshoot of the control system corresponding to the optimal results for algorithms 1, 2, and 3 was 14.3807%, 20.2146%, and 19.1002%, respectively. For higher requirements in stability of the control system, the penalty function *P*(*X*) can be modified, which will reduce the accuracy requirements simultaneously.

## 4. Conclusion

Under the same experimental conditions, an improved genetic algorithm was proposed in this work to improve the convergence speed, accuracy, and the probability to converge to the optimal value. The performance of the proposed algorithm had been verified by eight different kinds of typical test functions. Furthermore, the improved genetic algorithm had been applied to the parameter tuning of PID controller for liquid level controlling of beer filling machine, which revealed the superiority in effectively improving the rapidity of the control system with the premise of steady-state error elimination.

## Figures and Tables

**Figure 1:** Schematic diagrams of test function.

**Figure 2:** The average convergence curves of different algorithms.

**Figure 3:** The unit step response curve of the control system.

**Figure 4:** Bode plot of control system.

**Figure 5:** Convergence curves of different algorithms with equation (20) as the fitness function.

**Figure 6:** The unit step response curve of the control system with equation (20) as the fitness function.

**Figure 7:** Convergence curves of different algorithms with equation (22) as the fitness function.

**Figure 8:** The unit step response curve of the control system with equation (22) as the fitness function.

**Table 1:** Comparison of average convergence precision of different algorithms.

Test function	Algorithm 1	Algorithm 2	Algorithm 3
Test function 1	0	6.9713 × 10^−12^	9.8716 × 10^−13^
Test function 2	5.8970 × 10^−11^	3.8843 × 10^−5^	4.0453 × 10^−5^
Test function 3	0	2.7837 × 10^−3^	4.0595 × 10^−3^
Test function 4	0	3.8579 × 10^−1^	3.3787 × 10^−1^
Test function 5	0	8.4037 × 10^−5^	3.4528 × 10^−4^
Test function 6	0	3.4295 × 10^−3^	1.0409 × 10^−3^
Test function 7	2.1673 × 10^−11^	2.0123 × 10^−3^	1.5920 × 10^−4^
Test function 8	0	1.5393 × 10^−3^	4.8283 × 10^−3^

**Table 2:** Comparison of average convergence algebras of different algorithms.

Test function	Algorithm 1	Algorithm 2	Algorithm 3
Test function 1	88	159	160
Test function 2	21	59	62
Test function 3	56	152	161
Test function 4	110	200	200
Test function 5	88	181	197
Test function 6	111	196	195
Test function 7	63	121	136
Test function 8	75	175	160

**Table 3:** Comparison of probability of convergence to the optimal value of different algorithms.

Test function	Algorithm 1	Algorithm 2	Algorithm 3
Test function 1	100	81	87
Test function 2	97	55	45
Test function 3	100	67	57
Test function 4	100	55	52
Test function 5	100	43	49
Test function 6	100	83	82
Test function 7	94	60	57
Test function 8	100	50	46

**Table 4:** Comparison of performance indexes of control system with equation (20) employed as the fitness function.

Performance indexes	Before PID correction	Algorithm 1	Algorithm 2	Algorithm 3
Steady-state error, *e*_ss_	0.1669	0	0	0
Adjustment time, *t*_*s*_	96.7520	12.7310	16.3020	16.4000
Overshoot, *σ*(%)	0	71.9570	102.3144	108.0654

## Data Availability

The data used to support the findings of the study can be obtained from the author upon request.
